# Effect of Combining Operating Room Nursing Based on Clinical Quantitative Assessment with WeChat Health Education on Postoperative Complications and Quality of Life of Femoral Fracture Patients Undergoing Internal Fixation

**DOI:** 10.1155/2022/2452820

**Published:** 2022-02-09

**Authors:** Qingyan Liu, Juan Wang, Jie Han, Daiying Zhang

**Affiliations:** The Operating Room, The Affiliated Hospital of the Southwest Medical University, 25 Taiping Road, Luzhou City 646000, Sichuan Province, China

## Abstract

**Objective:**

To explore the effect of combining operating room nursing based on clinical quantitative assessment with WeChat health education on postoperative complications and quality of life (QOL) of femoral fracture patients undergoing internal fixation.

**Methods:**

Ninety femoral fracture patients treated in our hospital (July 2018 to July 2021) were chosen as the research objects and split into the control group (routine intervention) and the study group (combination of operating room nursing based on clinical quantitative assessment and WeChat health education) according to the nursing intervention modes, with 45 cases each. After nursing, the postoperative complications and QOL of patients were compared between the two groups.

**Results:**

No statistical between-group differences in general data were observed (*P* > 0.05); the hospital stay, weight-bearing time, and fracture healing time were obviously shorter in the study group than in the control group (*P* < 0.05); 1 d after surgery, the VAS pain status was not significantly different between the two groups (*P* > 0.05), and 2 d and 3 d after surgery, the VAS scores were significantly lower in the study group than in the control group (*P* < 0.05); 1 d after surgery, the Harris scores of patients in the two groups were close and did not present statistical difference (*P* > 0.05), and 8 weeks after surgery, the Harris score was significantly higher in the study group than in the control group (*P* < 0.05); the scores on self-care agency such as self-concept, self-care skills, sense of self-care responsibility, and health knowledge level were significantly higher in the study group than in the control group (*P* < 0.05); compared with the control group, the probability of occurring incision infection, lung infection, pressure sore, swelling and pain, and other complications was significantly lower in the study group (*P* < 0.05).

**Conclusion:**

Implementing operating room nursing based on clinical quantitative assessment combined with WeChat health education to femoral fracture patients undergoing internal fixation can effectively improve their postoperative clinical indicators, reduce their postoperative pain sensation and complication incidence, and effectively promote the joint motion range, which is conducive to enhancing their self-care agency and QOL.

## 1. Introduction

The femur is the largest bone in the whole body, and if femoral fracture is not treated promptly, it can trigger major bleeding, nerve damage, and other complications. In the acute clinical treatment period, debridement, reduction, and fixation of the fracture site should be performed. At present, internal fixation is one of the common procedures for femoral fracture reduction, but the high tension on the fracture end, premature weight-bearing exercise, and other reasons often lead to bending and breaking of intramedullary pins in patients and then the failure of internal fixation; in addition, intraoperative traction and postoperative fracture end reduction require adduction of the hip joint, which can easily trigger complications such as pudendal nerve palsy in patients. Also, as an invasive procedure, internal fixation can cause systemic stress responses and affect the postoperative recovery effect [1–4]. Therefore, the exploration of effective operating room nursing is of great importance for smooth surgery and reducing patients' stress responses. The quantitative assessment strategy has been introduced in the clinical practice of our hospital, which has provided reliable basis for the establishment and implementation of clinical nursing plan, and can effectively avoid many nursing risks caused by routine operating room nursing, standardize perioperative nursing work, and facilitate the implementation of safety management system, with significant clinical application effect. In recent years, with the development of high-tech technologies, such as artificial intelligence and sensing technology, medical services have also gradually moved into the real intelligence and promoted the development and flourishing of medical careers, and intelligent medical nursing has also been gradually spreading into more ordinary households [5–8]. Hence, by establishing a WeChat education platform, our hospital tried to carry out continuous nursing interventions to promote the nursing level and guarantee nursing quality for femoral fracture patients, with better clinical application effect. Currently, there are fewer studies related to combining operating room nursing based on clinical quantitative assessment with WeChat health education in orthopedic diseases, so 90 femoral fracture patients treated in our hospital were selected as the study objects to explore the effect of the combination of the two in postoperative complications and quality of life (QOL) in femoral fracture patients undergoing internal fixation.

## 2. Study Methods

### 2.1. Patients' Screening

The inclusion and exclusion criteria were decided according to the study objective. Inclusion criteria were as follows: ① all patients were diagnosed with femoral fracture after imaging examination; ② patients had complete medical data; ③ patients met the indications of internal fixation; ④ patients did not have history of surgical treatment; and ⑤ patients and their family members were aware of the study and signed the informed consent. Exclusion criteria were as follows: ① patients were complicated with severe organ and tissue lesion, coagulation disorder or malignancy; ② patients had pathological fracture; ③ patients had cognitive disorder, seeing-hearing disorder, or language disorder that affected chief complaint; ④ patients were complicated with other orthopedic diseases; ⑤ patients could not go along with the WeChat health education; and ⑥ patients had the history of fracture diseases or limb movement disorder. A total of 90 femoral fracture patients treated in our hospital from July 2018 to July 2021 were screened as the study objects.

### 2.2. Patients' Grouping

According to the nursing intervention modes, 90 patients were divided into the control group (routine intervention) and the study group (combination of operating room nursing based on clinical quantitative assessment and WeChat health education), with 45 cases each. The study was reviewed and approved by the Hospital Ethics Committee.

## 3. Methods

Control group: routine operating room nursing was performed, including preoperative routine examination, preparing surgical devices, paying close attention to the changes in patients' vital signs, maintaining patients' body temperature and room temperature, and assisting the doctors to finish the surgery; after surgery, routine nursing measures were carried out according to the patients' condition changes, and routine education (mainly one-on-one verbal communication) was conducted to patients and their family members; after discharge, regular telephone follow-up was performed to understand the recovery status of patients [9–12].

Study group: based on the above, operating room nursing based on clinical quantitative assessment combined with WeChat health education was performed. (1) Preoperative clinical quantitative assessment: patients' clinical data including BMI, age, Evans–Jensen classification, Self-Rating Anxiety Scale (SAS) score, bone quality, anemia, complications, and surgical anesthesia method were recorded for the clinical quantitative assessment, and each dimension was rated on a scale of 1–3 points; see Table 1. According to the results of the clinical quantitative assessment, graded nursing was performed; that is, those with the quantitative assessment score <10 points had low surgical risk; 10–13 points, medium risk; and >13 points, high risk. For the allocation of the nursing personnel, see Table 2. (2) Operating room nursing: ① before surgery, nursing personnel introduced the environment and medical staff of the operating room to the patients to reduce their sense of unfamiliarity of the operating room, alleviate their inner fear and anxiety about the surgery, and enhance their confidence [13, 14]. ② When performing the internal fixation to femoral fracture patients, the patients should be kept in a special position (lithotomy position) by traction, so during the surgery, the nursing personnel should assist the patients to keep in such position, pay close attention to the patients' changes in vital signs including heart rate, breath, and blood pressure, and pacify patients with encouraging words or actions to perform anesthesia. ③ During surgery, the nursing personnel should keep the room temperature at 23–26°C and the humidity at 50–60%, perform transfusion to patients according to the medical advice and maintain their body temperature, and assist the doctors to complete surgical operation. ④ After surgery, the nursing personnel paid timely attention to the patients' condition, cleared the surgical devices, conducted scientific pain management after the patients were awake by distracting them in the form of communication, massage, etc., and took analgesic measures in case of severe pain according to the medical advice. (3) Perioperative WeChat health education: first, a WeChat group consisting of physician-in-charge, special nurses, head nurse, and primary nurse was established. After admission, routine health education was performed to patients, including disease introduction, psychological intervention, related knowledge of perioperative period, functional exercise, and discharge guidance; after the patients joined the WeChat group, the medical personnel informed the patients and their family members of the objective and effect of setting the WeChat group and guided them to learn relevant knowledge, and the medical staff in the WeChat group were available for answering questions and consultation 24 h a day; according to the content modules and sequence of femoral fracture introduction, preoperative prevention and treatment of complications, preoperative functional exercise, surgical method introduction, preoperative preparation, self-adjustment of emotions, postoperative 6 h status, functional exercise, diet guidance, and discharge guidance, and in the form of WeChat video, posters and pictures, texts, and audio explanation, the nursing personnel pushed the health knowledge to the WeChat group.

### 3.1. Observation Indicators

Patients' general data including age, BMI, gender, affected side, Evans–Jensen classification, complications, and educational level were recorded. During clinical nursing, patients' hospital stay, weight-bearing time, and fracture healing time were recorded.

Patients' pain status was assessed by visual analogue scale (VAS), a visual scale marked with 0–10 for the patients to make judgement according to their pain sensation, with “0” indicating “no pain,” “10” indicating “unbearable severe pain,” and the numbers in between referring different degrees of pain. The physician assigned a score according to the position marked by the patients, and in clinical evaluation, 0–2 points indicated excellent, 3–5 points indicated good, 6–8 points indicated fair, and >8 points indicated poor. Three days after surgery is a critical period when patients experience frequent pain, and the pain will gradually disappear with fracture healing, and therefore, patients' pain was assessed at 1 d, 2 d, and 3 d postoperatively.

After surgery, patients' hip joint mobility was assessed by the Harris Hip Scale (HHS), which covered four domains, pain, function, absence of deformity, and range of motion (ROM). The maximum score was 100 points, and the results could be interpreted with the following: >90 = excellent, 80–89 = good, 70–79 = fair, and <70 = poor. Fracture healing is a long process. The assessment of patients' hip joint motor function 1 d after surgery was used as the baseline data, and 8 weeks after surgery, the basic morphology of fracture healing could be seen, and therefore, patients' hip joint motor function and healing status were assessed.

Patients' self-care agency was assessed by the Exercise of Self-Care Agency (ESCA) scale [15], which contained self-concept, self-care skills, sense of self-care responsibility, and health knowledge level and had 48 items. Each item was rated with the 5-grade scoring method (1–5 points), and the score for each dimension was the average score of items of such dimension, with higher scores indicating stronger self-care agency. The scale had Cronbach's *α* coefficient of 0.88 and retest reliability of 0.65.

Patients' QOL level after intervention was assessed by World Health Organization Quality of Life (WHOQOL)-BREF [16] from the aspects of psychology, physiology, environment, and social relations, and the score of each domain was obtained by the mean score of item of such domain multiplied by 4, with higher scores indicating better QOL. Cronbach's *α* coefficient of WHOQOL-BREF was 0.90, the Guttman split-half reliability coefficient was 0.86, and Cronbach's *α* coefficients in the field of physiology, psychology, society, and environment were, respectively, 0.74, 0.72, 0.72, and 0.87. After surgery, patients' complications were recorded.

### 3.2. Statistical Processing

In this study, the between-group differences in data were calculated by SPSS 22.0, the picture drawing software was GraphPad Prism 7 (GraphPad Software, San Diego, USA), the items included were enumeration data and measurement data, which were expressed by *n*(%) and ±*s* and examined by the chi-square test and *t*-test, respectively, and differences were considered statistically significant at *P* < 0.05.

## 4. Results

### 4.1. General Data

No statistical between-group differences in general data including age, BMI, gender, affected side, Evans–Jensen classification, complications, and educational level were observed (*P* > 0.05). See Table 3.

### 4.2. Basic Clinical Indicators

Compared with the control group, the patients' hospital stay, weight-bearing time, and fracture healing time were obviously shorter in the study group (*P* < 0.05). See Table 4.

### 4.3. Pain Status

One day after surgery, the difference in VAS pain status of patients in the two groups was not significant (*P* > 0.05), and 2 days and 3 days after surgery, the VAS scores were significantly lower in the study group than in the control group (*P* < 0.05). See Figure 1.

### 4.4. Joint Mobility

One day after surgery, the Harris scores of the two groups were close and did not present statistical difference (*P* > 0.05), and 8 weeks after surgery, the Harris score was significantly higher in the study group than in the control group (*P* < 0.05). See Figure 2.

### 4.5. Self-Care Agency

Compared with the control group, the study group obtained significantly higher self-care agency scores on self-concept, self-care skills, sense of self-care responsibility, and health knowledge level (*P* < 0.05). See Table 5.

### 4.6. QOL

The WHOQOL-BREF scores on psychology, physiology, environment, and social relations were obviously higher in the study group than in the control group (*P* < 0.05). See Figure 3.

### 4.7. Complications

Compared with the control group, the study group had significant probability of occurring incision infection, lung infection, pressure sore, swelling and pain, and other complications (*P* < 0.05). See Table 6.

## 5. Discussion

Femoral fractures are mostly caused by trauma and often present with pain, swelling, altered shape of the affected limb, functional impairment, etc., seriously affecting patients' normal life. Currently, the internal fixation and reduction in broken bone by instruments are the main treatment modality for such patients, and internal fixation can promote healing for performing early functional exercises and effectively reduce the occurrence of various complications. As the medical technology is advancing, the treatment methods and effects of femoral fractures have been significantly improved, but iatrogenic factors are still important factors affecting the patient outcome at present, with operating room nursing being the main component [17–20]. With the abundant resource of femoral fracture patients undergoing internal fixation, our hospital had rich experience in operating room nursing and found that routine operating room nursing placed emphasis on the doctor's procedure with the main purpose of assisting the doctor to finish the procedure, and so did the clinical practice, so routine operating room nursing was passive and limited to some extent and could not meet the gradually increasing nursing needs from current social and medical development. The clinical quantitative assessment strategy is the condition quantitative assessment scale generated on the basis of the evidence-based medicine and evidence level, which can fully consider the individual situation of patients and carry out multidimensional evaluation to perform systematic nursing intervention according to the physiological and psychological status of patients, making clinical nursing more scientific, comprehensive, and efficient [21–24]. To further improve the clinical nursing level of our hospital, WeChat health education was implemented for femoral fracture patients during the perioperative period, which promoted the intensity of nursing intervention and obviously improved patients' psychological state, self-care ability, etc. Based on this, some femoral fracture patients undergoing internal fixation treated in our hospital were selected as the study objects to explore the effect of combining operating room nursing based on clinical quantitative assessment with WeChat health education on postoperative complications and QOL of such patients.

The study concluded that compared with the control group, the patients in the study group had obviously shorter hospital stay, weight-bearing time, and fracture healing time (*P* < 0.05), which was consistent with the report by Chen et al. [25], proving that combining operating room nursing based on clinical quantitative assessment with WeChat health education effectively improved patients' postoperative recovery effect and significantly promoted nursing quality. In addition, the incidence rates of postoperative complications were significantly lower in the study group than in the control group (*P* < 0.05), indicating that the combined intervention greatly reduced the postoperative stress responses in femoral fracture patients undergoing internal fixation and thus obviously lowered the complication incidence. Preoperative quantitative assessment of patients' BMI, age, anemia, complications, and other clinical data is mainly to deeply understand their body status, realize surgical risk grading with intuitive and scientific quantitative data, and create more complete and comprehensive surgical plan, which is beneficial for reducing intraoperative accidental trauma. The joint application of WeChat health education intervention is conducive to increasing the degree of patients' perception of the disease and surgery and reducing their psychological burden. Therefore, the combination of the two will adjust the patients' physical and mental status to the best, fundamentally guaranteeing smooth operation.

By rating the surgical risks of patients through clinical quantitative assessment, patients' nursing needs can be intuitively embodied, and the allocation of nursing personnel conducted on this basis fully reflects the timeliness and pertinence of operating room nursing. In addition, WeChat health education during the perioperative period increases the nurse-patient bonding and elevates the trust between nurses and patients. As the study objects were mostly elderly people with insufficient perception of their physical function and disease cognition, combining operating room nursing based on clinical quantitative assessment with WeChat health education could make up for the two aspects and had better application effect in taking precautions against surgical risks and performing psychological intervention for patients in particular. The study concluded that 1 d after surgery, the VAS pain status was not significantly different between the two groups (*P* > 0.05), and 2 d and 3 d after surgery, the VAS scores were significantly lower in the study group than in the control group (*P* < 0.05); 1 d after surgery, the Harris scores of patients in the two groups were close and did not present statistical difference (*P* > 0.05), and 8 weeks after surgery, the Harris score was significantly higher in the study group than in the control group (*P* < 0.05); the scores on self-care agency such as self-concept, self-care skills, sense of self-care responsibility, and health knowledge level were significantly higher in the study group than in the control group (*P* < 0.05); and the WHOQOL-BREF scores on psychology, physiology, environment, and social relations were obviously higher in the study group than in the control group (*P* < 0.05). Based on patients' pain assessment and joint function, operating room nursing based on clinical quantitative assessment combined with WeChat health education could promote postoperative recovery by reducing postoperative stress responses and elevating disease perception, and the combination effectively reduced patients' pain symptoms, improved patients' joint function to some extent, and promoted their QOL.

In conclusion, the implementation of operating room nursing based on clinical quantitative assessment combined with WeChat health education for femoral fracture patients undergoing internal fixation can effectively improve their postoperative clinical indicators, alleviate their postoperative pain sensation, reduce their postoperative complications, benefit the promotion of their self-care ability and QOL, and also greatly improve their joint ROM. As this study was a retrospective analysis study with a small sample size and a single center, subsequent related studies should expand the sample size to confirm the conclusion herein; in addition, intelligent medicine is evolving, and the WeChat health education model applied in this study still has great potential for promotion, which can be explored in depth in subsequent studies to form a more complete WeChat education scheme.

## Figures and Tables

**Figure 1:** Between-group comparison of VAS scores. Note: the horizontal axis showed the time points, and the vertical axis showed the score; one day, two days, and three days after surgery, the VAS scores of the control group were 8.67 ± 0.35, 6.52 ± 0.38, and 5.67 ± 0.42, respectively; one day, two days, and three days after surgery, the VAS scores of the study group were 8.56 ± 0.41, 5.48 ± 0.34, and 4.11 ± 0.39, respectively; ^*∗*^ indicated significant between-group difference in VAS scores 2 days after surgery (*t* = 13.682, *P* < 0.001); ^∗∗^ indicated significant between-group difference in VAS scores 3 days after surgery (*t* = 18.258, *P* < 0.001).

**Figure 2:** Between-group comparison of the Harris scores. Note: the horizontal axis denoted the time points, and the vertical axis denoted the score; one day and eight weeks after surgery, the Harris scores of the control group were 43.14 ± 2.81 and 80.27 ± 3.36, respectively; one day and eight weeks after surgery, the Harris scores of the study group were 43.25 ± 2.50 and 91.88 ± 2.15, respectively; ^*∗*^ indicated significant difference in Harris scores 8 weeks after surgery between the two groups (*t* = 19.524, *P* < 0.001).

**Figure 3:** WHOQOL-BREF scores of the two groups. Note: the horizontal axis presented the assessment dimensions, and the vertical axis presented the score; the WHOQOL-BREF scores on psychology, physiology, environment, and social relations of the control group were 12.25 ± 1.76, 13.06 ± 2.37, 12.03 ± 2.18, and 11.20 ± 2.54, respectively; the WHOQOL-BREF scores on psychology, physiology, environment, and social relations of the study group were 14.05 ± 1.55, 14.21 ± 2.30, 13.44 ± 2.25, and 13.25 ± 2.57, respectively; ^*∗*^ from left to right indicated significant differences in WHOQOL-BREF scores on psychology, physiology, environment, and social relations between the two groups (*t* = 5.149, 2.336, 3.019, and 3.806, *P* < 0.001, = 0.022, = 0.003, and <0.001).

**Table 1:** Preoperative clinical quantitative assessment.

Evaluation item	1 point	2 points	3 points
BMI (kg/m^2^)	Normal	Underweight or overweight	Fat
Age (years)	<70	70–79	>79
Evans–Jensen classification	I	II-III	IV
SAS score (points)	<60	60–69	>69
Bone quality	Normal	Osteopenia	Osteoporosis
Anemia	None	Mild	Moderate and above
Complications	None	1	2 and above
Anesthesia method	Nerve block	Intravertebral anesthesia	General anesthesia

**Table 2:** Graded nursing.

Allocation of nursing personnel	Low risk	Medium risk	High risk
Work experience <3 years/advanced nurse	1	0	1
3–5 years of work experience/nurse	1	1	1
Work experience >5 years/supervisor nurse	0	0	1

**Table 3:** General data of the two groups (*n* = 45).

Observation indicator	Control group	Study group	*X* ^2^/*t*	*P*
Age (years)	70.85 ± 10.12	71.26 ± 10.43	0.189	0.850
BMI (kg/m^2^)	20.15 ± 4.33	20.08 ± 4.29	0.077	0.939
Gender (male/female)	23/22	25/20	0.044	0.833
Affected side (left/right)	24/21	22/23	0.045	0.833
Evans–Jensen classification				
I	10 (22.22)	8 (17.78)	0.278	0.598
II	16 (35.56)	15 (33.33)	0.049	0.824
III	14 (31.11)	15 (33.33)	0.051	0.822
IV	5 (11.11)	7 (15.56)	0.385	0.535
Complications				
Diabetes mellitus	3 (6.67)	2 (4.44)	0.212	0.645
Coronary heart disease	4 (8.89)	3 (6.67)	0.155	0.694
Hypertension	6 (13.33)	7 (15.56)	0.090	0.764
Osteoporosis	10 (22.22)	12 (26.67)	0.241	0.624
Anemia	13 (28.89)	14 (31.11)	0.053	0.818
Others	9 (20)	7 (15.56)	0.304	0.581
Educational level			0.046	0.830
Junior high school and below	26 (57.78)	27 (60)		
Junior high school and above	19 (42.22)	18 (40)		

**Table 4:** Basic clinical indicators.

Group	Hospital stay (d)	Weight-bearing time (d)	Fracture healing time (weeks)
Control	18.45 ± 3.17	62.71 ± 6.55	12.84 ± 1.08
Study	12.86 ± 3.05	56.39 ± 6.12	10.55 ± 0.89
T	8.524	4.729	10.977
P	<0.001	<0.001	<0.001

**Table 5:** Scores on self-care agency of the two groups.

Group	*N*	Self-concept	Self-care skills	Sense of self-care responsibility	Health knowledge level
Control	45	3.44 ± 0.55	3.26 ± 0.57	3.36 ± 0.57	3.51 ± 0.61
Study	45	3.95 ± 0.48	3.80 ± 0.45	3.64 ± 0.55	3.85 ± 0.42
*T*		4.687	4.988	2.391	3.080
*P*		<0.001	<0.001	0.020	0.003

**Table 6:** Occurrence of complications of the two groups (*n*(%)).

Complication	Control group	Study group	*X* ^2^	*P*
Incision infection	2 (4.44)	0 (0)		
Lung infection	2 (4.44)	0 (0)		
Pressure sore	5 (11.11)	2 (4.44)		
Swelling and pain	5 (11.11)	2 (4.44)		
Others	4 (8.88)	1 (2.22)		
Total incidence rate	18 (40)	5 (11.11)	9.870	0.002

## Data Availability

Data that support the findings of this study are available on reasonable request from the corresponding author.
